# Drug-Induced Deafness: A Rare Case of Bilateral Sensorineural Hearing Loss Following Speedballing

**DOI:** 10.7759/cureus.20686

**Published:** 2021-12-25

**Authors:** Zaheer Ahmad Qureshi, Elina Shrestha, Pravash Budhathoki, Haider Ghazanfar, Arundhati Dileep, Muhammad S Akhter

**Affiliations:** 1 Internal Medicine, Icahn School of Medicine at Mount Sinai, New York, USA; 2 Internal Medicine, BronxCare Health System, Bronx, USA; 3 Internal Medicine, Continental Medical College, Lahore, PAK; 4 Nephrology, BronxCare Health System, Bronx, USA

**Keywords:** sudden sensorineural hearing loss, recreational drug use, speedballing, heroin abuse, cocaine use

## Abstract

Many users of recreational drugs use cocaine and opioids together, often called “speedballing.” Hearing loss is a rarely reported adverse effect following recreational drug abuse. Only one case has been reported in history with hearing loss caused by speedballing. Here, we present the case of a 38-year-old female who presented with speedball abuse and new-onset bilateral hearing loss to the emergency department. A computed tomography scan of the head was unremarkable. She was treated with thiamine, folate, multivitamins, and intravenous fluids. The hearing loss improved without any acute intervention. The significance of sudden hearing loss due to recreational drug use is highlighted by this case. Apart from a few animal studies, there is no detailed research explaining the pathophysiology of speedball-induced hearing loss. Further studies and trials are needed to better understand the effects of combined and separate cocaine and opioid use on audiologic physiology.

## Introduction

Although rare, auditory disorders, including sensorineural hearing loss following recreational drug use, have been linked to cocaine and opioids, especially heroin. Some of the known psychiatric and neurological side effects of cocaine include anxiety, schizophrenia, and neurovascular deficits [1]. Significant cardiovascular effects are caused by stimulation of the sympathetic nervous system. Heroin is a central nervous system depressant and may lead to coma, respiratory arrest, and stroke [2]. Many people use cocaine and heroin together, called a speedball. It produces a heightened sense of euphoria if used combined compared to either drug alone. There are some reports of hearing loss associated with cocaine or heroin but rarely together.

In some cases, cochlear implantation for auditory rehabilitation is required. Little is known regarding the effects of cocaine and heroin together, especially on the ear. The goal of this report is to describe a case of bilateral sensorineural hearing loss following speedballing.

## Case presentation

A 38-year-old female presented to the emergency department after being found unresponsive at her home with pinpoint pupils and decreased respiratory rate. She was accompanied by her male friend who stated that she had consumed alcohol and snorted some unknown substance in her nose. The patient confessed to drinking alcohol and taking cocaine before losing a sense of what was happening. On initial examination, she had a new-onset bilateral hearing loss, more prominent in the left ear than the right ear, also associated with vertigo. She heard a loud “whooshing sound” and could not hear anything else afterward. She complained of dizziness but denied any history of ear pain, ear discharge, ear ringing, nausea, vomiting, vision change, or weakness. She had no history of trauma to her ears. She has no significant medical history. Her surgical history was also unremarkable. She used to live alone in her apartment. She was an occasional smoker, consumed beer once a week, and had been using illicit substances such as cocaine and heroin on weekends for a long time.

She was hypoxic in the field and was administered bag valve mask ventilation which increased her oxygen saturation to 100%. Her blood glucose level was 51 mg/dL. She was given 0.5 mg of Narcan intravenously plus 2 mg intranasally and became responsive with blood glucose level improving to 183 mg/dL. In the Emergency Department, she had tachycardia (110 beats per minute), but the rest of her vitals were stable. Her laboratory investigations at the time of admission are presented in Table 1.

**Table 1:** Results of the initial blood workup.

Blood workup	Results
Sodium	134 (135–145mEq/L)
Potassium	4.6 (3.5–5.0 mEq/L)
Serum chloride	99 (98–108 mWq/L)
Serum bicarbonate	15 (24–30 mEq/L)
Serum glucose	89 (70–120 mg/dL)
Blood urea nitrogen	14 (0.5–1.5 mg/dL)
Creatinine	1.4 (0.5–1.5 mg/dL)
Total serum calcium	7.5 (8.5–10.5 mg/dL)
Phosphorus	7.4 (2.5–4.5 mg/dL)
Serum magnesium	2.1 (1.5–2.7 mg/dL)
Total bilirubin	0.2 (0.2–1.2 mg/dL)
Direct bilirubin	<0.2 (0.0–0.3 mg/dL)
Total serum protein	7.3 (6.0–8.5 g/dL)
Serum albumin	3.9 (3.2–4.8 g/dL)
Alanine aminotransferase	1,915 (5–40 U/L)
Aspartate transaminase	2,447 (9–48 U/L)
Gamma-glutamyl transferase	26 (8–54 U/L)
Serum creatine kinase	180 (20–200 U/L)
Serum alkaline phosphatase	68 (42–98 U/L)
Serum acetaminophen	<5 (10.0–30.0 ug/mL)
Serum acetylsalicylic acid	<0.3 (3.0–10.0 mg/dL)
Serum ethanol	<10 (≤10 mg/dL)
Serum ammonia	37 (11–35 µmol/L)
Prothrombin time	11.6 seconds (27.2–39.6 seconds)
Partial thromboplastin time	28.5 seconds (9.9–13.3 seconds)
International normalized ratio	1.01 (0.85–1.14)
Urine drug screen	
Cocaine	Positive
Cannabinoid	Negative
Benzodiazepine	Negative
Methadone	Negative
Opiate	Negative
Phencyclidine	Negative
Arterial blood gas analysis	
pH	7.21(7.350–7.450)
Partial pressure of carbon dioxide	55.4 mmHg (35.0–45.0 mmHg)
Partial pressure of oxygen	37.4 mmHg (83.0–108.0 mmHg)

An electrocardiogram revealed sinus tachycardia. Chest X-ray and computerized tomography scan of the head were unremarkable. She was admitted to the Intensive Care Unit. On physical examination, there were no external ear injuries, her bilateral eardrums were intact, and there was no blood or injury in the external auditory canal. Neurological examination revealed no abnormalities, and Romberg’s sign was negative. The patient was treated with thiamine, folate, multivitamins, normal saline, and famotidine. Otolaryngology (ENT) was consulted for hearing loss. On examination, she was found to have bilateral hearing loss, which was more prominent in the left ear. Furthermore, ENT advised a formal hearing test in the ENT lab. The poison control center was consulted for overdose and supportive care was advised.

Her urine drug screening was positive for cocaine. Anti-nuclear antibody, viral hepatitis, and anti-mitochondrial antibodies were negative; however, anti-smooth muscle antibody was positive. Her hearing loss improved to the baseline on its own the next day, and she was transferred to the medical floor. Subsequently, the patient’s liver function tests downtrended. The subsequent ENT evaluation two days after her admission revealed no hearing abnormalities, and the patient was planned for outpatient audiogram evaluation. She eloped from the hospital and has been lost to follow-up on subsequent attempts to reach her.

## Discussion

Cocaine is an alkaloid that is produced from the *Erythroxylum coca* plant. The standard routes of administration are nasal insufflation, smoke inhalation, or intravenous, with nasal insufflation having the highest bioavailability of 80% [3]. It is a stimulant that binds to the receptors of neurotransmitters and blocks their uptake, thereby increasing the concentration of dopamine, norepinephrine, and serotonin in the synapses. The reinforcing properties of cocaine are primarily due to the enhancement of dopamine transmission in the mesocorticolimbic dopamine pathway. An increase in dopamine at the synapses activates the G protein intracellular signaling pathways leading to the phosphorylation of transcriptional factors. This increases the excitability of the prefrontal cortex, which is thought to be the changes caused by cocaine [4]. Cocaine is also a potent vasoconstrictor due to its alpha-adrenergic agonism [3]. Fandino et al. conducted a study in rabbits and demonstrated that endothelin-1 mediated the cerebral vasospasm caused by cocaine [5]. It is also a local anesthetic due to its alteration in the neuronal sodium channels [6].

Hearing loss after cocaine use is an uncommon event, and more research is yet to be done to understand the exact mechanisms causing the effect. Shivapuja et al. conducted a cocaine injection experiment on Chinchillas. They found decreased inner ear cochlear blood flow likely due to the inhibition of the reuptake of norepinephrine at the synaptic cleft leading to vasoconstriction [7]. Heinz et al. conducted studies in baboons after injecting intramuscular cocaine. They found that cocaine impaired the discrimination of tones and speech sounds. They suggested cocaine’s interference with the central nervous system’s processing of the acoustic cues [8].

Although several case reports have been published regarding hearing loss after cocaine use, only one case report has been published reporting speedball-induced hearing loss [9]. Nicoucar et al. presented a case of unilateral hearing loss in the left ear after intranasal ingestion of cocaine along with alcohol. They found intralabyrinthine hemorrhage of the ear, diagnosed using magnetic resonance imaging. The vascular effects of cocaine were thought to be the cause [10]. Fowler et al. reported a case of sudden-onset bilateral sensorineural hearing loss after speedballing with cocaine and heroin. The absence of otoacoustic emissions in the transient evoked otoacoustic emissions and elevated acoustic reflexes in the audiogram confirmed cochlear and neural components, respectively [9]. Ciorba et al. presented a case of sudden-onset bilateral hearing loss after intravenous injection of cocaine. Audiometry revealed symmetrical sensorineural hearing loss and transitory evoked otoacoustic emissions (TEOAEs) were absent on both ears. The patient had complete restoration of hearing after treatment with betamethasone. Additionally, they discussed the possibility of cocaine altering or blocking the K+ channels of the inner hair cells and suggested that the cochlear damage was due to the perturbation of cochlear homeostasis rather than reduced blood supply [11]. Stenner et al. published a case of sudden-onset bilateral sensorineural hearing loss without vestibular deficits after intravenous cocaine injection. The absent TEOAEs confirmed the presence of significant cochlear pathology. They found that the higher frequencies were affected severely. The patient had a normal return of hearing by day three of hospitalization, and the patient was treated with prednisone and pentoxifylline. They suggested the cause to be related to the reduced blood supply [12]. Opioid abuse can lead to deafness. Although the pathophysiology of opioid-associated hearing loss is unclear; numerous theories have been proposed. Two of the common theories are ischemic cochlear secondary to vasospasm or vasculitis and the direct effect of opioids on opioid receptors [13].

In our case, the patient likely used some form of opiate, which was not detected in the urine toxicology screen, as she was responsive after Narcan injection. However, the urine toxicology was only positive for cocaine. There is a high probability that the patient used speedball, a combination of cocaine and opioids, especially heroin. Our patient had all the signs and symptoms (pinpoint pupils, unconsciousness, and respiratory depression) of the opioid overdose triad [14]. She also responded immediately to Narcan which further increased the clinical suspicion that she might have used a combination of cocaine and opioids. Another indicator the patient might have used opioids was her history of heroin use. Our patient was unsure if she took anything besides cocaine. Our patient had a normal ENT evaluation after two days of presentation. She did not receive any specific therapy for her hearing loss, as used in the other case reports. She only received thiamine, folate, multivitamins, and intravenous fluids. Except for a few animal model experiments, there is no detailed research explaining the pathophysiology related to speedball-induced hearing loss. More studies are required to better understand the pathophysiology.

## Conclusions

Our case highlights the significance of recreational drug use leading to sudden hearing loss. Apart from a few animal model experiments, there is no detailed research explaining the pathophysiology of speedball-induced hearing loss. A physician should keep this complication in mind while treating patients with recreational drug use. Further studies and trials should be conducted to better understand the effects of cocaine and opioids combined and when used separately on audiologic physiology.
